This article has been retracted.

# Biomolecular Modulation of Neurodegenerative Events during Ageing

**DOI:** 10.1155/2015/978654

**Published:** 2015-10-25

**Authors:** Marcella Nebbioso, Gianfranco Scarsella, Aloisa Librando, Nicola Pescosolido

**Affiliations:** ^1^Department of Sense Organs, Sapienza University of Rome, Piazzale Aldo Moro 5, 00185 Rome, Italy; ^2^Department of Biology and Biotechnology Charles Darwin, Sapienza University of Rome, Piazzale Aldo Moro 5, 00185 Rome, Italy; ^3^Department of Cardiovascular, Respiratory, Nephrology, Geriatric, and Anesthetic Sciences, Sapienza University of Rome, Piazzale Aldo Moro 5, 00185 Rome, Italy

## Abstract

The objective is to assess the modulation of retinal and optic nerve degenerative events induced by the combination of *α*-lipoic acid (ALA) and superoxide dismutase (SOD) in an animal model of ageing. For this study, 24 male Wistar-Harlan strain rats were left to age for up to 24 months. One group of rats was subjected to a diet supplemented with ALA and SOD for 8 weeks, while another group was used as a positive control and not subjected to any dietary treatment. To assess the cytoprotective effects of the antioxidants, a morphological analysis was carried out on sections of retina and optic nerve head, stained with haematoxylin-eosin, followed by an analysis of the modifications to nuclear DNA detected by the TUNEL technique. The lipid peroxidation assay was used to assess the damage induced by oxidative stress at cell membrane level. The molecules involved in apoptosis mediated by oxidative stress, such as caspase-3 and inducible nitric oxide synthase, were also assayed by immunolocalization and western blot. ALA and SOD are able to counteract senile neurodegenerative deterioration to the retina and optic nerve. Indeed, the combination of these antioxidant molecules can reduce oxidative stress levels and thus prevent both nuclear degradation and subsequent cell death.

## 1. Introduction

The term oxidative stress was first coined in 1989 by Sies who defined it as an imbalance between the production of free radical species and antioxidant defence systems [1]. In physiological conditions, the inside of the cell has a negative charge owing to an array of enzymes and molecules that counterbalance its production. Moreover, the cells of all aerobic organisms produce most of their chemical energy by consuming oxygen in their mitochondria. Mitochondria are thus the main place where intracellular oxygen consumption is the major source of reactive oxygen species (ROS) formation [1, 2]. Alongside ROS, there is a family of free radicals that affects the type of nitrogen known as reactive nitrogen species (RNS), which includes nitric oxide (NO). The enzyme responsible for the production of NO in cells is nitric oxide synthase (NOS), present in three isoforms. It is capable of catalysing the conversion of the amino acid L-arginine into L-citrulline, with the release of NO [3]. Two of the three isoforms of NOS, the constitutively expressed brain and endothelial NOS, are dependent on concentrations of calcium and calmodulin and generate limited amounts of NO. The third isoform of NOS, also known as inducible nitric oxide synthase (iNOS), is calcium independent, not found in the tissues under normal conditions, and produces such high amounts of NO that it induces cytotoxicity [3, 4]. The expression of iNOS was detected in optic nerve astrocytes in patients with glaucoma, a disease that causes increased intraocular pressure (IOP) and ischaemia of the optic nerve [3]. As the body grows older, in accordance with the theory of ageing, normal antioxidant levels are no longer sufficient to counteract the generation of free radicals (FR) [5]. The increase in FR causes molecular damage, some of it being irreversible that accumulates in tissues with age [5, 6]. Nohl and Hegner (1978) were the first to observe that there is greater production of superoxide radical in the liver of 19-month-old than in that of 6-month-old rats [7].

It has been shown that retinal tissue is particularly susceptible to oxidative damage. Indeed, it is one of the most metabolically active tissues in the body, contains an abundant number of mitochondria, and is subjected to constant photochemical stress [8]. For these reasons, ocular nerve cells are able to produce high concentrations of radical species which, if not sufficiently neutralized, can cause multiple incidents of oxidative damage to the hydrocarbon chains of unsaturated fatty acids, to the amino acid residues of proteins, to the nitrogenous bases of nucleic acids, and to carbohydrates [8].

In extreme cases, all this can be followed by alteration and functional impairment of all the structures, leading to cell death. The death of a significant number of retinal ganglion cells (RGCs) also leads to a reduction in the number of axons forming the optic nerve. The evolution of this phenomenon causes functional deterioration of the optic nerve, which eventually results in neurosensory visual deficit [9].

To counteract this oxidative damage, the body has at its disposal a series of antioxidants that, even at very low concentrations, are able to delay or inhibit oxidation of the substrate [10]. One of the major enzyme systems involved in this defence is superoxide dismutase (SOD), a ubiquitous enzyme that plays a key role in the defence mechanisms against the ROS and RNS produced during cellular metabolism [11]. Some foods containing SOD include melon, wheat sprouts, maize, and soybeans. SOD catalyzes the dismutation of the superoxide anion into hydrogen peroxide and molecular oxygen. In mammals, there are three isoforms of SOD expressed by cells: copper- and zinc-containing SOD (CuZnSOD or SOD1) is a homodimer primarily localized to the cytoplasm; manganese SOD (MnSOD or SOD2) is a homotetramer localized exclusively in the mitochondrial matrix and is found in multiple organisms; and extracellular SOD (ECSOD or SOD3) shares significant amino acid homology with CuZnSOD (40–60%) and contains both copper and zinc in its active site but is localized to the extracellular region of the cell. Each isoform is a product of distinct genes and with distinct subcellular locations, but catalyses the same reaction [11].

Several studies using knockout mice have shown that mitochondrial MnSOD (mitSOD) is essential for survival. Indeed, mice lacking this isoform exhibit various symptoms such as damage to the myocardium and liver, lipid peroxidation, and mitochondrial dysfunction and do not survive for more than three weeks. Conversely, where the cytosolic Cu/ZnSOD isoform is missing, mice appear normal and exhibit abnormalities only after trauma [12].

Conversely, increased SOD production in transgenic or mutant strains of* Caenorhabditis elegans* and* Drosophila melanogaster* leads to increased tolerance to oxidative stress and therefore longevity [13, 14].

A second line of defence is also formed by endogenous antioxidant compounds, including *α*-lipoic acid (ALA), a water-fat-soluble vitamin derivative, isolated for the first time in 1951 from bovine liver [15]. Humans can only synthesize small amounts of ALA from fatty acids and cysteine, so they need exogenous substances [16–18]. ALA is found primarily in animal sources such as liver, heart, muscle, and kidney. To a lesser extent it is also present in fruits and vegetables: broccoli, spinach, tomatoes, potatoes, and rice bran [16–18]. ALA is regarded as a scavenger of free radicals; it has two oxidized or reduced thiol groups and is able to neutralize various reactive species of ROS and RNS. ALA also has the ability to greatly increase intracellular glutathione (GSH) levels, as well as hepatic levels of ascorbate, which conversely decline with age [19, 20].

Based on these considerations, we decided to undertake an experimental study to evaluate the ability of ALA and SOD to modulate the physiological phenomena of ocular neurodegeneration linked to ageing and caused in large part by the damaging effects of the production and accumulation of free radicals. To this end, the study used an experimental animal model in order to reproduce the biochemical and histopathological framework typical of cellular ageing.

## 2. Materials and Methods

### 2.1. Animals and Treatments

All experimental procedures were in accordance with the ARVO Statement for the Use of Animals in Ophthalmic and Vision Research, the guidelines of the European Communities Council Directive of 24 November 1986 (86/609/EEC), Italian Health Ministry guidelines, and EU Directive 2010/63/EU for animal experiments.

Twenty-four male Wistar-Harlan rats, aged between 20 and 24 months (centenarian rats) with an average weight of 300 to 350 g, were divided into two groups. The first group of rats was pretreated with the same diet for eight weeks, supplemented with ALA and SOD, while the second group was used as a positive control and was not subjected to any supplementary treatment. The dosage of the product per kilogram of body weight was equal to 8.57 mg/day for ALA and 2 IU/day for SOD, that is, corresponding to the human diet, equal to 600 mg/day of ALA and 140 IU/day of SOD (ALA600 SOD, Alfa Wassermann, Bologna, Italy). The negative control group was made up of 12 young male rats of the same strain, aged between 4 and 6 months, and with an average weight of 200 to 250 g, fed normally. The animals were then sacrificed by carotid bleeding, after which the eyeballs were removed.

### 2.2. Experimental Procedures

The degenerative process was assessed using morphological techniques, immunohistochemistry, western blot, and lipid peroxidation (LPO) assays. The aim was to find morphological, nuclear, and cell membrane damage both at retinal and at optic nerve level. Cytotoxicity and apoptotic markers were also assessed.

### 2.3. Molecular Analysis of Tissue Sections and of Retina Total Protein Extracts: Morphology Techniques and Sample Preparation

The eyes were enucleated, the corneas were rapidly cut vertically, and the crystalline lens and vitreous humour were removed. We then carried out the following procedures on the residual tissues: fixation in paraformaldehyde 4% for 6 hours at 4°C; rapid wash with 1X PBS pH 7.4; immersion in a 30% sucrose solution in 1X PBS pH 7.4 at 4°C overnight; and embedding in Killik embedding medium (Bio-Optica, Milan, Italy) in order to perform the cryostat cut into 10 *μ*m sections, horizontally, to allow longitudinal observation of the optic nerve. The sections were placed on microscope slides and stored at −20°C.

In order to observe their morphology, the samples were stained with haematoxylin-eosin. The sections, left to dry at room temperature, were subjected to the following treatments: rehydration with decreasing alcohol (100°, 95°, and 75°) for 7.5 minutes; distilled water for 5 minutes; haematoxylin 0.1% for 1 minute (to stain the chromatin); running water for 10 minutes; distilled water for 2 minutes; eosin for 45 seconds (to stain cytoplasmic components); distilled water for 2 minutes; dehydration with increasing alcohol (75°, 95°, and 100°) for 7.5 minutes; and mounting of the slides with glycerol-PBS 1 : 3. Finally, the tissue sections were observed under an optical microscope and photos taken using computerized image acquisition.

### 2.4. TUNEL Assay

Tissue sections with a thickness of 10 *μ*m were subjected to TUNEL technique (Terminal deoxynucleotidyl transferase mediated dUTP Nick End Labeling). It consists of* in situ* labelling of DNA fragments by fluoresceinated nucleotide conjugation using terminal deoxynucleotidyl transferase, iNOS, and caspase-3. At an advanced stage of the apoptosis cascade, the cell presents extensive DNA degradation which leads to the production of molecules 180–200 bp in length and their multiples.

The sections, left to dry at room temperature for 30 min, were subjected to the following treatments: rehydration through a descending alcohol series (100°, 95°, and 75°, 2 min each); incubation with protease 20 *μ*g/mL in Triton X-100 to 0.1% at 37°C for 30 min; washes with 1X PBS for 2 min; incubation with the TUNEL reagent (*In Situ* Cell Death Detection Kit, AP, ROCHE), containing 1/10 in volume of terminal deoxynucleotidyl transferase and the remaining fraction of nucleotides labelled with a fluorescent chromophore, 10 *μ*L per section at 37°C for 1 h. On each slide, one of the sections was always used as the negative control, that is, incubated only with the nucleotides but without terminal transferase in order to detect any nonspecific staining of the sections; washes with 1X PBS for 5 min; and mounting of the slides with Eukitt. The observations were made under a fluorescence microscope and pictures taken by computerized image acquisition.

### 2.5. Lipid Peroxidation (LPO) Assay

The LPO-586 assay was used to assess the presence of oxidative stress at cell membrane level. This technique is based on the reaction of two molecules of the chromogenic reagent, N-methyl-2-phenylindole (R1), with one molecule of malondialdehyde (MDA) at 45° to form a stable chromophore with maximum absorbance at 586 nm. LPO-586 is a detection kit distributed by* Bioxytech*. Normally, in this kit there is an* insert system* to avoid several experimental problems. The retinas were collected from the enucleated eyes, weighed, transferred to a glass tube with 230 *μ*L of* lysis buffer*, and homogenized in a glass-glass* Potter homogenizer* to carry out the LPO assay. The samples were then subjected to three freeze-thaw cycles and then added to 650 *μ*L of diluted R1 reagent and then 150 *μ*L of HCl (12 N). Subsequently, the samples were incubated at 45°C for 60 minutes and centrifuged at 15000 ×g for 10 minutes. The supernatant was collected in a cuvette to measure absorbance at 586 nm. The blank sample was prepared in the same manner, but with the addition of acetonitrile (75%) and diluent (25%) and not diluted R1. Standard data were used to calculate the absorbance of each sample by subtracting the blank value from the values measured in the spectrophotometer at 586 nm. The MDA concentration was calculated from the absorbance value by linear regression analysis.

### 2.6. Fluorescence Immunolocalization

This method was used to locate iNOS and caspase-3 in the retina and optic nerve head. iNOS is one of the main molecules induced in the case of tissue damage, while caspase-3 is the protease responsible for the final stages of the apoptotic cascade. To detect iNOS and caspase-3 expression we used primary polyclonal anti-iNOS and anti-caspase-3 antibodies (Santa Cruz) produced in rabbits (diluted to 1 : 50 and 1 : 100, resp.) while the secondary antibodies used were goat anti-rabbit IgG Alexa Fluor antibodies (Molecular Probes) that are green-fluorescing. The sections, left to dry at room temperature for 30 min, were subjected to various treatments: washes in 1X PBS for 5 min; postfixation with alcohol at increasing volumes (70°, 95°, and 100°) for 2 min; washes in 1X PBS for 5 min; block with serum (NRS or NGS), 10% in PBS, 1 h in a moist chamber; incubation with the primary antibody diluted in 1X PBS and BSA 1% for 1 h; fast washes in 1X PBS; incubation with the secondary antibody diluted 1 : 200 in 1X PBS and 1% of the serum of the animal in which the antibody was produced, for 30 min at room temperature; washes in 1X PBS for 5 min; and mounting of the slides with Eukitt. The observations were made under a fluorescence microscope and pictures taken by computerized image acquisition.

### 2.7. Western Blotting and Immunodetection

Western blotting was used for the identification and quantization of iNOS and caspase-3 on retinal protein extracts. The results were normalized by locating *α*-tubulin, constitutively expressed in the cells. The Bradford assay was then used to extract protein from animal tissues and to estimate their concentration, by measuring the absorbance at 595.0 nm of IGg, at known increasing concentrations, to which the Bradford reagent was added. Measuring the absorbance of these standards provided a calibration line, on which the protein sample concentration was calculated. The proteins were then subjected to electrophoretic separation on SDS-PAGE (SDS-*Polyacrylamide Gel Electrophoresis*). After weighing the tissues, they were immersed in lysis buffer, and the protein was extracted. The test-tubes were kept for 10 min on ice both before and after centrifugation, performed twice at 13000 rpm for 5 seconds. Subsequently, the supernatant was collected to be used in the study.

*Solutions and Gels. Upper gel buffer 4x* is as follows: Tris/Cl, pH 6.8, 0.5 M, and SDS 0.4%.* Lower gel buffer 4x* is as follows: Tris/Cl, pH 8.8, 1.5 M, and SDS 0.4%.* Stacking gel* is as follows: upper gel buffer 2.5 mL H_2_O 6.6 mL, acrylamide solution 30% 1.1 mL, APS (ammonium persulfate) 10% 100 *μ*L, and TEMED (tetramethylethylenediamine) 10 *μ*L.* Resolving gel* (*12%*) is as follows: lower gel buffer 2.5 mL, H_2_O 4.1 mL, acrylamide solution 30% 4.1 mL, APS 10% 50 *μ*L, and TEMED 5 *μ*L.* Loading buffer* (*10 mL*) is as follows: 18% glycerol, 2% SDS, 2.5% bromophenol blue, 5% *β*-mercaptoethanol, 2.5 mL stacking gel buffer 4x, and H_2_O to volume.* Gel running buffer 1x* is as follows: 25 mM Tris base (3 g/L), 192 mM glycine (14.4 g/L), and 0.1% SDS, all titrated to pH 8.3.

### 2.8. Transfer of Proteins to Nitrocellulose

The transfer took place by pressing the gel against a nitrocellulose filter in a constant 300 mA electric field. The filter was then washed with T-TBS 1X 0.1% and after saturation of nonspecific bonds (T-TBS 1X + milk 5%), the proteins were probed with the primary antibody capable of specifically detecting those of interest. The same antibodies were used as for the immunolocalization of iNOS and caspase-3. Normalization was performed by recognizing *α*-tubulin (goat, Santa Cruz) and the anti-tubulin antibody was diluted 1 : 1000, while all others were diluted 1 : 500. During incubation, each antibody was added to a solution of T-TBS and dry milk 5% for one hour. After several washes with T-TBS, carried out following absorption of the primary antibody, incubation with the secondary antibody was performed. The secondary antibodies used for caspase-3 and iNOS (*anti-rabbit* IgG,* Jackson*) and *α*-tubulin (*anti-goat IgG, Jackson*) were used at a dilution of 1 : 5000. Finally, detection by electrochemiluminescence (ECL) was performed.

*Solutions and Products. Blotting buffer 1X* is as follows: 25 mM Tris base (3 g/L), 192 mM glycine (14.4 g/L), 20% methanol.* T-TBS 1X 0.1%*, 5 mM Tris/Cl pH 7.4, 15 mM NaCl, and 0.1% Tween 20.* Blocking buffer 1x* is as follows: T-TBS 1X 0.1% and dry milk 5% final.

### 2.9. Statistical Analysis

All the experiments were repeated at least four times. Statistical analysis of results was made by the ANOVA test. Significativity of result was evaluated by Student's *t*-test. Followed by Student's *t*-test, *p* values < 0.05 were considered significant.

## 3. Results

### 3.1. Morphology of the Retina and Optic Nerve Head

Cryostat sections of experimental and control rat eyes were stained with haematoxylin-eosin. Any changes in the astrocyte cells were observed, as well as any morphological changes to the retinal layers and changes to the nuclear chromatin.

Tissue sections from the eyes of young rats not subjected to treatment showed no abnormalities (Figure 1(a)) but were used to highlight the alterations in the optic nerve head of aged rats.

In tissue sections from the eyes of control aged rats not treated with antioxidants, there was a reduction in neural tissue due to apoptosis of RGCs and loss of optic nerve axons and apoptosis of astrocytes (Figure 1(b)). The main alteration it was possible to highlight was the thinning of the optic nerve head following ageing.

In the tissue sections from aged rats treated with ALA- and SOD-based antioxidants, a smaller papillary loss and a good columnar shape typical of astrocyte cells were highlighted (Figure 1(c)).

### 3.2. Study of Modifications due to DNA Degradation (TUNEL Assay)

This technique labels the nucleus of cells in an advanced stage of death, where endonucleases have fragmented the DNA. Nuclei with degraded DNA showed greater fluorescence than nuclei in which the degenerative process was absent, because the terminal transferase specifically incorporates fluorescent nucleotides onto the free 3′OH ends of fragmented DNA (Figures 2(a) and 2(b)). Indeed, in the sections of guinea-pig eye pretreated with ALA and SOD (Figure 2(c)), the assay was not very positive, due to reduced degradation of DNA caused by the cytoprotective effect of the antioxidants both on the astrocyte cells and on the RGCs.

### 3.3. Study of Modifications to Cell Membranes (LPO-586 Assay)

The oxidative stress induced an increase in membrane damage. The extent of membrane damage was assessed by measuring the production of MDA, a widely recognized marker of lipoperoxidation whose production occurs in cells as a direct result of damage to the membrane structure and function. Samples obtained from aged rats showed very high cytoplasmic MDA concentrations with extensive lipoperoxidative damage. By contrast, treatment with ALA and SOD reduced levels of all apoptosis markers, as well as improving overall homeostatic response and limiting apoptotic phenomena (Figure 3).

### 3.4. Immunolocalization of iNOS and Caspase-3

There was no immunolocalization of iNOS in juvenile rats, while the cells of normal-fed aged rats had high iNOS expression (Figures 4(a) and 4(c′)). High cytotoxic levels of NO were then detected. Conversely, immunofluorescence was reduced in the sections of aged rats fed with ALA and SOD, indicating reduced expression of iNOS (Figures 4(c) and 4(c′)). This would confirm that this enzyme is activated in the presence of damage caused by ageing, as in our model (Figures 4(b), 4(c), 4(b′), and 4(c′)).

Similarly, no significant activation of caspase-3 was observed in juvenile rats (Figures 5(a) and 5(c′)). Conversely, significant expression of caspase-3 was found (indicating suffering and therefore apoptotic activation and the consequent cell death induced by ageing) in sections of eyes from untreated aged rats (Figures 5(b) and 5(b′)), whereas in rats fed with ALA and SOD there was a marked decrease in the expression of this protease (Figures 5(c) and 5(c′)).

### 3.5. Western Blot Analysis of iNOS and Caspase-3

The iNOS band was less present, as confirmed by western blot in aged rats pretreated with ALA and SOD (Figure 6), as seen previously via immunolocalization. As expected, a decrease in caspase-3 expression was also observed in retinal extracts subjected to antioxidant treatment, indicating that the reduction in cell death was due to lower activation of the apoptotic death programme (Figure 6). Normalization was performed using the expression of *α*-tubulin, constitutively expressed in the cells. In both cases, the bands obtained from the different samples were subjected to quantization by ECL and the values obtained were expressed as percentages (Figure 7 and Table 1).

## 4. Discussion

The primary aim of our work was to use an experimental animal model to reproduce and assess the histological and therefore biochemical phenomena of cell ageing. Secondarily, we investigated the changes of antioxidant molecules, such as ALA and SOD, on the harmful effect of the free radicals that accumulate over the normal biological processes of life.

From the various parameters considered, we observed that the antioxidant combination of ALA and SOD, administered for 8 weeks to aged rats, would be able to counteract the degenerative events associated with ageing. In fact, our assays seem to confirm that older and therefore damaged tissues have significant iNOS expression. Once NO is produced, it is capable of causing irreversible damage to tissues [21–23]. The toxicity of iNOS has been found in several inflammatory and degenerative eye diseases such as multiple sclerosis, Parkinson's disease, and Alzheimer's disease [22, 23]. Studies of iNOS overexpression in mice have shown that increased NO levels would be able to cause the apoptotic death of retinal photoreceptors [24]. Furthermore, our study would seem to highlight the fact that a reduction in NO, through the use of antioxidants, could provide significant therapeutic benefits against the retinal degeneration induced by oxidative stress due to natural causes, such as ageing. Presumably, the positive effect could also follow a cell degeneration with various pathological causes such as inflammatory, traumatic, or metabolic disorders [17, 18, 22, 25, 26].

Furthermore, the increased stability of mitochondrial membranes, as demonstrated by the reduction in the LPO reaction induced by free radicals, would help reduce the release of proapoptotic factors responsible for inducing the programmed cell death process.

Interestingly, in some studies, it has been found that changes in mitochondrial membrane permeability can lead to opening of transition pores (PTPs) in the liver and brain of aged rats. This would lead to the subsequent release of cytochrome c [27]. Cytochrome c, when released into the cytoplasm, interacts with Apaf-1 to form a protein complex called the apoptosome, which promotes activation of caspase and therefore of the apoptotic death cascade [28].

Going forward, Kokoszka et al. have shown that chronic oxidative stress in mice leads to a partial deficiency in MnSOD which would entail an increase in the sensitization of mitochondrial PTPs and consequently induce apoptosis [29]. Indeed, SOD, as well as MnSOD in particular, plays a major role in maintaining normal mitochondrial function and structural integrity [30]. It has been found that mutant mice totally lacking MnSOD suffer from severe mitochondrial defects, mainly in the brain and heart [12, 31, 32].

Furthermore, differential expressions have been shown to exist between the Bcl-2 family of proteins and the caspase family during ageing in the rat brain [25, 33]. Data confirm these studies, indicating that aged rats would show a marked expression of caspase-3, an executioner protease known to take part in the final stages of the apoptotic cascade [34]. Thus, the oral administration of ALA and SOD would also reduce the activation of this protease, thereby preventing the apoptotic death of retinal cells and the consequent loss of axons forming the optic nerve.

ALA is regarded as one of the most important antioxidants and therefore has an equally significant therapeutic value in pathological conditions related to the overproduction of radicals with oxidative capacity. Furthermore, its reduced form, dihydrolipoic acid, reacts by neutralizing such radicals as superoxide, hydroxyl radicals, hypochlorous acid, peroxides, and singlet oxygen [35, 36].

Some Authors have observed that ALA reduces the markers of apoptosis and oxidative stress more significantly than SOD. But these effects seem particularly relevant when treatment is administered concomitantly with ALA and SOD, probably due to the presence of synergistic mechanisms of action. Mainly, SOD acts in the extracellular environment, and conversely ALA also acts in intracellular level [4, 14, 18, 26].

## 5. Conclusion

In summary, this study appears to show that, during the RGC ageing process, axons in the optic nerve cells and astrocytes are subjected to an array of degenerative damage, due mainly to an increase in oxidative stress levels. The damage would no longer be countered by the normal antioxidant defence systems which, as is known, decline with age. Oral administration of ALA and SOD would provide a number of significant benefits against the retinal degeneration mediated by oxidative stress. This is due to a reduction in DNA fragmentation and iNOS expression caused by antioxidants' ability to counteract the high levels of free radicals typical of ageing. This would thus improve the condition of treated eye nerve tissue compared with control cases. Furthermore, the lower LPO assay obtained from the antioxidant combination would improve membrane integrity, thus protecting retinal cells and optic nerve fibres from tissue death.

Ultimately, further research will be required in order to gain a better understanding of the different ways in which antioxidants act, not only in advanced stages of life but also in the course of pathological events with inflammatory, tumoral, traumatic, and dystrophic causes.

## Figures and Tables

**Figure 1:** Morphology of the retina and optic nerve head stained with haematoxylin-eosin. (a) Section of the optic nerve head of a young rat with no obvious abnormalities (6 months, negative control). (b) Section of the optic nerve head of an untreated aged rat (24 months, positive control). The main alteration it was possible to highlight was the increased excavation of the optic nerve head. (c) Section of the optic nerve head of an aged rat after oral supplementation with *α*-lipoic acid (ALA) and superoxide dismutase (SOD) (24 months, positive control). Here, a smaller papillary excavation and a good columnar shape typical of astrocyte cells were highlighted compared to the section in panel (b).

**Figure 2:** Modifications to nuclear DNA (*TUNEL assay*). (a) Section of the optic nerve head of a young rat with no obvious abnormalities (6 months, negative control). (b) Section of the optic nerve head of an untreated aged rat (24 months, positive control). Nuclei with degraded DNA showed greater fluorescence than nuclei in which the degenerative process was absent. (c) Section of the optic nerve head of an aged rat after oral supplementation with *α*-lipoic acid (ALA) and superoxide dismutase (SOD) (24 months, positive control). In this case, the assay was not positive, due to reduced degradation of DNA caused by the cytoprotective effect of the antioxidants.

**Figure 3:** Level of membrane lipoperoxidation (LPO) in retina samples and role of *α*-lipoic acid (ALA) and superoxide dismutase (SOD) in the control of apoptosis. Bars report the level of malondialdehyde (MDA) evaluated as indicated in the following legend for each bar. The values represent mean ± S.E.M. Controls = young rats (untreated); positive rats = aged rats (untreated); positive rats ALA + SOD = aged rats after treatment with ALA and SOD.

**Figure 4:** Inducible nitric oxide synthase (iNOS) immunolocalization in the sections of the optic nerve head (a/b/c) and in the retina (a′/b′/c′). ((a) and (a′)) Young rat without iNOS immunolocalization (6 months, negative control). ((b) and (b′)) Aged rat fed normally with high iNOS expression in cells. ((c) and (c′)) Aged rat after oral supplementation of *α*-lipoic acid (ALA) and superoxide dismutase (SOD) with reduced immunofluorescence, indicating lower iNOS expression.

**Figure 5:** Caspase-3 immunolocalization in the sections of the optic nerve head (a/b/c) and in the retina (a′/b′/c′). ((a) and (a′)) Young rat without caspase-3 immunolocalization (6 months, negative control). ((b) and (b′)) Aged rat fed normally with high caspase-3 expression. ((c) and (c′)) Aged rat after oral supplementation of *α*-lipoic acid (ALA) and superoxide dismutase (SOD) with reduced immunofluorescence, indicating lower caspase-3 expression.

**Figure 6:** Western blot analysis of inducible nitric oxide synthase (iNOS) and caspase-3. (1) Young rats. (2) Untreated aged rats: increased presence of iNOS and caspase-3 bands. (3) Treated aged rats: iNOS and caspase-3 bands are less frequent.

**Figure 7:** Quantization of the inducible nitric oxide synthase (iNOS) and caspase-3 bands obtained by western blot. The iNOS and caspase-3 were less present in aged rats pretreated with antioxidants indicating that the reduction in cell death was due to lower activation of tissue damage and apoptotic death.

**Table 1:** The inducible nitric oxide synthase (iNOS) and caspase-3 bands in the different samples were subjected to quantization by electrochemiluminescence (ECL) and the values obtained were expressed as a percentage.

Bands	(A) Aged rats Untreated	(B) Aged rats ALA + SOD treated	(C) Young rats Controls	(A)-(B) *p*	(B)-(C) *p*
iNOS	100%	26 ± 4	6 ± 2	**≤0.01** ^**∗**^	≤ 0.1
Caspase-3	100%	23 ± 3	8 ± 2	**≤0.01** ^**∗**^	≤ 0.1

Mean values ± SD. Significativity of the results was considered with ^*∗*^ *p* values < 0.05.

## Abbreviations

ALA: *α*-Lipoic acid
SOD: Superoxide dismutase
LPO: Lipid peroxidation
iNOS: Inducible nitric oxide synthase
ROS: Reactive oxygen species
RNS: Reactive nitrogen species
RGCs: Retinal ganglion cells
NO: Nitric oxide
NOS: Nitric oxide synthase
IOP: Intraocular pressure
FR: Rree radicals
CuZnSOD or SOD1: Copper- and zinc-containing SOD
MnSOD or SOD2: Manganese SOD
ECSOD or SOD3: Extracellular SOD
mitSOD: Mitochondrial MnSOD
GSH: Glutathione
TUNEL: Terminal deoxynucleotidyl transferase mediated dUTP Nick End Labeling
R1: Methyl-2-phenylindole
MDA: Malondialdehyde
SDS-PAGE: SDS-polyacrylamide gel electrophoresis
APS: Ammonium persulfate
TEMED: Tetramethylethylenediamine
ECL: Electrochemiluminescence
PTPs: Permeability of transition pores.
